# A Systematic Review of Lymphangioleiomyomatosis on Diagnosis and Molecular Mechanism

**DOI:** 10.1155/2021/6612776

**Published:** 2021-02-10

**Authors:** Xiaotong Dong, Lvcheng Jin, Ailan Wang, Liping Wu, Xintong Fan, Qian Hou, Tianbao Li, Ruilian Zhao, Yunxiang Zhang

**Affiliations:** ^1^Department of Pathology, First Affiliated Hospital of Weifang Medical University, Weifang People's Hospital, Weifang 261041, China; ^2^Department of Science, Qingdao Geneis Institute of Big Data Mining and Precision Medicine, Qingdao, China; ^3^Department of Respiratory, First Affiliated Hospital of Weifang Medical University, Weifang People's Hospital, Weifang 261041, China; ^4^Department of General Practice, Affiliated Hospital of Weifang Medical University, Weifang 261031, China

## Abstract

**Objective:**

Lymphangioleiomyomatosis (LAM) is a rare low-grade metastatic tumor; however, LAM patients were always found in young age with difficulty for diagnosis. Our study is aimed at observing the clinical characteristics of patients with lymphangiomatosis, including the clinical manifestations, imaging findings, histopathological features, and immunophenotype.

**Methods:**

We did a systematic review on LAM/PLAM cases, especially on male cases, and collected the clinical features and molecular mechanisms of PLAM based on previous findings.

**Results:**

Diagnosis criteria were summarized by combining CT scans, MRI, immunohistochemistry results, and gene sequencing results for effectively distinguishing between PLAM and similar diseases. Moreover, our study illustrated the molecular mechanism of PLAM as well as the signaling pathway involved in the disease initials. In addition, a male case was reported with differential diagnosis on the clinical manifestations, microscopic features, immunophenotypes, and genotypes.

**Conclusion:**

Our review will definitely improve the understanding of diagnosis and treatment in PLAM cases.

## 1. Introduction

Lymphangioleiomyomatosis (LAM), a rare low-grade metastatic tumor, is classified as perivascular epithelioid cell tumor in the WHO lung tumor classification [1, 2]. Kitaichi et al. studied more than 300 patients. Their average age of onset was 35 years. The pathological findings showed that the normal lung parenchyma was replaced by multiple small cysts with a diameter of 0.1 several centimeters and there were signs of smooth muscle hyperplasia around and inside the pulmonary lymphatic vessels, veins, and airways [3]. The clinical manifestations of LAM at the onset are relatively mild, most of which are progressive dyspnea, often accompanied by spontaneous pneumothorax [4], cough, chylothorax, peritoneal effusion, and hemoptysis [5]. Pulmonary lymphangioleiomyomatosis (PLAM) and axial lymphatic cystic mass called tumor LAM can lead to abdominal and pelvic lymph obstruction [6]. Tuberous sclerosis (TSC) is an inherited tumor syndrome associated with epilepsy, cognitive impairment, and multiorgan tumor formation. It has been reported that LAM occasionally occurs in patients with TSC [7]. Studies have found that LAM is often associated with angiomyolipoma in the kidneys and can increase the incidence of meningioma [8]. The rate of lung function decline in LAM patients may be 2 to 4 times higher than that in ordinary people [9, 10]. Most patients will have difficulty in breathing in daily activities and recurrent pneumothorax within 10 years after the onset of symptoms [11]. The disease progression of LAM was not as fast as that of other cancers; however, clinical characteristics vary among patients. Respiratory failure was considered one of the main causes of the death in LAM patients; however, a prognostic approach for detecting respiratory failure has not been established [12].

At present, no specific cause of PLAM has been found and it is rare in male cases. Kazuhiro et al. reported a 17-year-old man with LAM after pneumothorax surgery. This patient was the youngest case reported, because histopathological diagnosis of pneumothorax in young men is not always possible; this case provides new and valuable clinical insights into pneumothorax in young men [13]. Another 22-year-old male patient with PLAM was reported to explore possible additional pathogenesis. The clinical, radiographic, and histopathological features of the patient were the same as those previously reported [14]. A 34-year-old man was diagnosed with a 2-year TSC and underwent transcatheter arterial embolization (TACE) for right renal hemorrhage caused by renal tumor. He was admitted to the hospital for frequent recurrent pneumothorax on the right side; chest computed tomography showed multiple small round, thin-walled cystic lesions in his both lungs. Recurrent pneumothorax is considered to be associated with PLAM disease with tuberous sclerosis (TSC-LAM). TSC-LAM is extremely rare; small bullae in early LAM may lead to missed diagnosis in some cases, so they are often diagnosed as spontaneous pneumothorax [15]. In high-resolution computed tomography (HRCT), a 37-year-old male patient had left pneumothorax and a large number of collapsed lungs with extensive parenchymal cysts in both lungs. This patient had normal phenotype and karyotype, suggesting that LAM may occur in normal male with unaffected TSC. Therefore, even if there is no sign of TSC, the possibility of LAM cannot be ruled out when a person has a diffuse cystic lung disease [16]. Kim et al. reported a man with PLAM and multiple hepatic angiomyolipoma, which led to the diagnosis of tuberous sclerosis. This unusual manifestation further broadens the clinical and pathological spectra of PLAM and hepatic angiomyolipoma. Therefore, the authors emphasized the distinction between multiple hepatic angiomyolipoma and hepatic tumor, while PLAM may be a cause of cystic lung disease even in a man [17]. Another report revealed a rare case of LAM in a male patient with tuberous sclerosis who developed pneumothorax after mechanical ventilation [18, 19]. Although these reports provide references for the diagnosis and treatment of PLAM, the specific causes of PLAM have not been discovered and few male patients have been reported. Therefore, there is an urgent need to understand the clinical manifestations and molecular mechanisms of PLAM in order to provide better diagnosis and treatment for patients.

In this study, we did a systemic review of LAM/PLAM disease in the aspects of diagnosis criteria and molecular mechanism. Furthermore, rare case of PLAM in male has been detailed presented with the clinical manifestations and immuno/genotypes serving as differential diagnosis reference for PLAM.

## 2. Diagnosis Criteria

In a clinical work, PLAM should be distinguished from the following diseases.

### 2.1. Idiopathic Pulmonary Fibrosis (IPF)

The imaging manifestations of both PLAM and IPF are characterized by diffusely distributed balloons of varying sizes, but the distribution of the gas-bearing cavities of the two is obviously different. PLAM is evenly distributed throughout the lung field, while IPF is mostly distributed in the middle and lower lung fields. Moreover, PLAM often has ground glass-like density shadows, consolidation shadows, subpleural arc shadows, and honeycomb shadows on CT images. The main pathological manifestations of IPF are a distorted alveolar structure and pulmonary interstitial fibrosis, in which inflammatory cells and fibroblast foci can be detected; the normally distributed lung tissue is scattered between the lesions, showing the coexistence of new and old lesions, which is obviously different from PLAM.

### 2.2. Benign Metastatic Leiomyoma

Benign metastatic leiomyoma mostly manifested as nodules in the lung parenchyma, with cystic changes in the nodules, but no cystic spaces.

### 2.3. Lymphangioma

Lymphangioma occurs in neonates and children. Under the microscope, the lymphatic vessels are dilated and the number is increased. It contains lymph fluid and lymphocyte nests, and the boundary is clear.

### 2.4. Lymphangiomatosis

Lymphangiomatosis is characterized by complicated hyperplasia of lymphatic vessels. Hyperplastic lymphatic vessels often invade the lung parenchyma, mediastinum, and chest wall and often have multifocal growth. Lymphocyte stones and complex proliferation of the maze can be seen under the microscope. They are lined with flat endothelial cells, and macrophages containing blood-side proteins can be seen in part of the lung cavity. Fine-needle aspiration biopsy is a rapid, economical, and minimally invasive pathological diagnosis technique with high sensitivity and specificity. Although PLAM is relatively rare, fine-needle aspiration biopsy can still effectively identify PLAM and similar diseases by combining CT scans, MRI, immunohistochemistry results, and gene sequencing results (Figure 1).

The main imaging manifestations of PLAM are multiple (>10) thin-walled balloon-containing lesions, round or round shaped, with clear boundaries [20]. As the lesion progresses, the cystic cavity can gradually expand. The imaging findings of this case were diffuse multiple lung-containing airbags, round or quasiround, unequal in size, and with clear boundaries, which were consistent with the typical performance of PLAM. The final diagnosis of PLAM depends on histopathological examination. The typical histological characteristics are that the lesions are mostly distributed along the bronchi, blood vessels, and subpleura and that the lungs are diffused with multiple cystic cavities [21]. The nodular lesions are often located in the cyst wall. It is composed of immature smooth muscle cells and perivascular epithelioid cells, namely, LAM cells. LAM cells are rich in cytoplasm and eosinophilic and can infiltrate blood vessels and lymphatic vessels, causing pulmonary hemorrhage. Although the pathological examination of this case was a puncture tissue, the histological performance was typical. Under the microscope, some alveoli were expanded and merged to form pulmonary bullae. The blood vessels and lymphatic vessels expanded. The naive smooth muscle cells in the lung interstitial showed nodular hyperplasia. The cytoplasm is rich and eosinophilic. Immunohistochemical detection of PLAM showed that immature smooth muscle cells were stained positive for SMA, vimentin, desmin, and PCNA and epithelioid-like cells were stained positive for HMB45. In addition, LAM cells also showed positive staining for ER, PR, Melan-A, and actin [22], of which about 55%~75% were positive in perivascular epithelioid cell tumors. Serum VEGF-D levels may be associated with the clinical manifestations of PLAM, and one study reported that patients with lymphatic involvement had higher VEGF-D levels than those without lymphatic involvement [23, 24]. Most women with LAM present with cystic lung disease, and most need lung biopsy to confirm the diagnosis. Patients with a level of serum VEGF-D higher than 800 ng/L can be diagnosed as having LAM, and up to 70% of patients may avoid unnecessary invasive examination, while about 30% of patients with cystic lung diseases still need a lung biopsy for diagnosis.

Only 7 cases have been reported in the literature. Schiavina et al. reported a 17-year-old man with LAM after pneumothorax surgery (Table 1). PLAM is composed of sporadic PLAM disease and TSC-LAM. TSC and PLAM have similar molecular pathogenesis. TSC is an inherited disease caused by TSC1 or TSC2 gene mutation. Adult female TSC patients with PLAM are quite common, with an incidence rate of up to 30%–40%; the estimated incidence of sporadic PLAM disease in adult women is about 1/400,000. However, male patients with PLAM are extremely rare. Patients with TSC should receive genetic counseling before pregnancy.

## 3. Molecular Mechanism

PLAM disease falls into two distinct types: some patients occur sporadically named S-LAM, and others are TSC-LAM [25, 26]. In recent years, our knowledge about the disease pathogenesis of PLAM has improved substantially. In either case of LAM, the major hallmark is mutational inactivation of tumor suppressor genes TSC1 and TSC2 encoding hamartin and tuberin protein, respectively [27–29]. For TSC-LAM patients, mutants within TSC genes usually occur in germ cells as well as in somatic tissues. In contrast, the results of one research indicated that somatic mutants rather than germline mutations were identified within the TSC1 or TSC2 gene in six of nine S-LAMSC1/TSC2 which were newly identified in PLAM patients by next-generation sequencing [30, 31]. PLAM is the most common lung manifestation of TSC and the third most common cause of TSC-related death. Due to de novo germline heterozygous mutations, about two-thirds of TSC-LAM cases have no family history of LAM [32]. Compared with the TSC-LAM type, S-LAM-type PLAM usually has more severe symptoms, starting at the age of 20-30 years, and the average age at diagnosis is later (about 35 years; TSC-LAM type is 30 years). What is more is that according to the patient's statement, the onset of the disease can be presumed until the age of 10, which is the youngest reported by the male PLAM whose parents and brothers are healthy. In addition, the sporadic type is more prone to LAM and other lymphatic vessel complications [33] and the deterioration of lung function is more serious. As we all know, lung function is closely related to the prognosis of PLAM, so the prognosis of the sporadic type is worse than that of the TSC-LAM type [32]. However, our current knowledge regarding additional functional molecules involved in PLAM disease is not enough to explicit phenotypic heterogeneity between S-LAM and TSC-LAM.

The genes TSC1 and TSC2 were located on chromosomes 9q34 and 16p13.3, respectively [34, 35], and the proteins hamartin and tuberin, respectively, which form heterodimeric complex TSC1/2 to interact with dozens of proteins. One of the interacting proteins named TBC1D7 and TSC1/2 heterodimer bind together to form the TSC1-TSC2-TBC1D7 complex (TSC-TBC) [36], which regulates the mammalian target of the rapamycin (mTOR) signaling pathway in response to upstream signals such as growth factor stimulation and hypoxia. That interaction process is not directly between TSC-TBC and mTOR but instead through suppressing the activity of an intermediate protein Ras homolog enriched in brain (Rheb) by the GAP domain of tuberin [37, 38]. Rheb is a member of the GTPases superfamily and is vital in the regulation of cell growth and cycle. mTOR is conserved serine-threonine kinase which constitutes the catalytic component of two complexes named Mtorc1 and Mtorc2. The other six components of mTORC1 were regulatory-associated protein of mTOR (Raptor), proline-rich Akt substrate of 40 kDa (PRAS40), mammalian lethal with Sec13 protein 8 (mLST8), telomere maintenance 2 (TELO2), TELO2-interacting protein 1 homolog (TTI-1), and DEP domain-containing mTOR-interacting protein (Deptor) [39, 40]. mTORC1 was involved in phosphorylation of a couple of target proteins including CLIP-170, Grb10, Lipin-1, ATG1, 4E-BP, and S6K, positively regulating cell proliferation by promoting microtubule organization, lipid glycerolipid metabolism, cell autophagy, and protein synthesis [41]. Blocking the mTORC1 pathway with S6K1 inhibitor gave rise to the failed phosphorylation of eIF4B, resulting in decreases of the translation efficiency of Fra1 and subsequent induction of the expression of the E-cadherin transcriptional repressor zinc finger E-box-binding homeobox 1/2 (ZEB1/2) [42]. ZEB1/2 is essential to induce the process of epithelial-to mesenchymal transformation (EMT) [43] which contributes to tumor cell migration and invasion. mTORC2 was comprised by eight subunits: five of them are the same as in mTOC1, and two components Raptor and PRAS40 were absent and substituted by mammalian stress-activated protein kinase-interacting protein (mSIN1), rapamycin-insensitive companion of mTOR (Rictor), and Proter [41]. mTOC2 plays important roles in cellular metabolism, cell survival, and proliferation as well as cytoskeleton organization by phosphorylating target proteins Rho, AKT [44], PKC [44], and SGK1 [45]. Stress fibre formation was altered by RhoA activity increasing through upregulation of mTORC2 and followed by cellular migration and cell survival increase [46] (Figure 2).

PLAM disease affects almost exclusively women, and especially, it is exacerbated during pregnancy when estrogen (E2) increased. One study has confirmed that the E2-ERK2 signaling pathway contributes to LAM pathogenesis [42]. E2 binds to its acceptor ER, and proto-oncogene tyrosine-protein kinase Src (c-Src) is phosphorylated by ER, and subsequent c-Src activates Ras. Activated Ras regulates the ERK pathway, in turn triggering kinase activity of proteins Raf, MEK, and ERK [47–49]. E2-stimulated ERK promotes RNA transcription of the Fra1 gene and phosphorylation of Fra1 protein, which in turn inducted ZEB1/2. ERK-ZEB1/2 is critical for the EMT process and to control cell proliferation, migration, and invasion. In addition, ERK upregulates the mTORC1 pathway by directly interacting with or repressing the TSC1/2 complex [47]. Therefore, when drugs targeted on both the E2-ERK and mTORC signaling pathways are combined, treatment for PLAM disease might be more effective. The LAM cells in this case were mainly immature smooth muscle cells with fewer epithelioid cells, so they did not express HMB45 and Melan-A. Other immunohistochemical results were vimentin (+), desmin (+), SMA (+), D2-40 (+), ER (individual+), PR (partial+), CK (epithelial+). Immunohistochemical characteristics are consistent with literature reports.

## 4. Discussion

In a comprehensive literature, PLAM usually occurs in females; the difference in the patients reported in this study was that the onset occurred in men; this case was the second reported case of male sporadic PLAM. These patient clinical manifestations were not obvious, the onset was earlier, and the history was long for more than 40 years. A male patient has been mistaken for having pneumonia many times, and only simple symptomatic treatment has been carried out. In the past 20 years, imaging examinations have shown slow progress and pathological examination has not been performed to confirm the diagnosis. He missed the best time for treatment and ultimately leading to a poor prognosis.

The male patient, 50 years old, was reported to have chest tightness, asphyxia, and other symptoms more than 40 years ago without obvious reasons or inducements, and his condition worsened after activity. After taking cough and anti-inflammatory drugs, he did not improve. Except that he could not perform heavy physical labor, other activities were not restricted. Because the abovementioned symptoms have become worse recently and there is a small amount of hemoptysis, the patient was suspected of having a mass in his lungs and was admitted to the Department of Respiratory Medicine. A physical examination was performed when the patient was admitted to the hospital. The patient was thin, lacked energy, and had irregular breathing and movement rhythms in both lungs, with widened intercostal spaces, low breath sounds. Abnormal results of other examinations are as follows: D-dimer of 51550.00 ng/mL, prothrombin time of 15.6 s, prothrombin activity of 56.00%, and prothrombin INR value of 1.36 INR. Chest CT showed multiple air-bearing thin-walled cysts in both lungs, which are round quasicircular, with clear boundaries. Compared with the CT results in 1998, there was no obvious progress. Percutaneous lung biopsy was performed after admission.

In this case, the patient was onset in adolescence. CT scan of his chest showed multiple thin-walled round well-defined air-filled cysts. The histopathological morphology was alveolar expansion, fusion with each other to form bullae, expansion of blood vessels and lymphatic vessels, immature smooth muscle cells in the lung interstitial nodular hyperplasia, abundant cytoplasm, and eosinophilic. Immunohistochemistry shows vimentin (+), desmin (+), SMA (+), D2-40 (+), ER (+), PR (+), CK (+), Melan-A (−), and HMB-45 (−). Sanger sequencing showed no TSC1/TSC2 gene mutation (Figure 3).

The puncture tissues were routinely dehydrated in 4% neutral formaldehyde solution, embedded with paraffin, then sliced, HE stained, and Congo red stained, and the morphology of the lesion was observed under a microscope. Immunohistochemical staining was performed using the EnVision method on a Roche BenchMark XT Ventana automatic staining machine. Staining procedures were setup strictly in accordance with the staining instructions for automatic immunohistochemical detection. Positive staining photos were set in each chip as required. Desmin, Melan-A, vimentin, SMA, D2-40, ER, PR, CK, HMB-45, CD68, S-100, and NSE antibodies are rabbit anti-human monoclonal antibodies (1 : 50; Beijing Zhongshan Jinqiao, China). We performed first-generation sequencing to detect whether there are TSC1/TSC2 gene mutations, we used the QIAamp DNA FFPE Tissue Kit to extract patient DNA, we amplified the target fragments by PCR, we detected the amplification results by agarose gel electrophoresis, and we used the ABI 3130XL sequencer to detect the presence of gene mutation. The diagnosis approach is as follows:

1. CT: the two lungs are filled with multiple gas-filled thin-walled cysts, which are round or round shaped, with varying sizes and clear boundaries (Figure 3(a1))
2. microscopic features: alveolar expansion and fusion to form pulmonary bullae, dilation of blood vessels and lymphatic vessels, and immature smooth muscle cells in the lung interstitial nodular hyperplasia; these cells are very rich in cytoplasm and eosinophilic (Figure 3(a))
3. immunohistochemistry and special staining: vimentin (+), desmin (+), SMA (+), D2-40 (+), ER (+), PR (+), CK (+), Melan-A (−), HMB-45 (−), CD68 (−), S-100 (−), NSE (−), and Congo red stain (−) (Figure 3(b))
4. generation sequencing: no TSC1/TSC2 gene mutation was detected in this case (Figure 3(c))
5. diagnosis: based on clinical manifestations, microscopic features, immunohistochemical staining, special staining, genetic testing, etc., combined with imaging features, this case can be diagnosed as PLAM
6. follow-up: the patient experienced sudden chest tightness and hemoptysis and was unable to lie down after a few hours of biopsy. There was no obvious pneumothorax on the chest radiograph. After active medical treatment, there was still repeated hemoptysis, low blood oxygen saturation, and respiratory failure. Due to severe lung lesions and a high risk of endotracheal intubation, the family of the patient refused to use endotracheal intubation ventilator-assisted ventilation treatment. The patient suddenly developed unconsciousness, respiratory arrest, and cardiac arrest symptoms on the second day after surgery. Rescue was invalid and clinical death was declared

In summary, the primary imaging findings of PLAM are multiple (>10) thin-walled balloon lesions, round or quasiround, with well-defined boundaries. As the lesion progresses, the cystic space gradually expands. The typical histological features are bronchial, vascular, and subcolumnar lesions, with multiple cystic cavities diffused in the lungs. Immunohistochemistry of PLAM showed that immature smooth muscle cells were positively stained for SMA, vimentin, desmin, and PCNA, while epithelial cells were positive for HMB45. In addition, serum VEGF-D levels may be related to the clinical manifestations of PLAM and LAM can be diagnosed in patients with serum VEGF-D levels higher than 800 ng/L. The final diagnosis of PLAM should be based on clinical manifestations, microscopic features, immunohistochemical staining, special staining, genetic testing, etc. Our systematic review focuses on the diagnosis and molecular mechanisms of LAM and PLAM, as well as a special case study, providing detailed instruction in clinical practice and improving the understanding of potential drug discovery.

## Figures and Tables

**Figure 1:** Tests for PLAM diagnosis process and criterion.

**Figure 2:** The signal pathway of the TSC1/2-TBC complex involved in PLAM.

**Figure 3:** Pathological diagnosis in our study case. (a) CT axial position (pulmonary window), showing multiple lung types with varying sizes of multiple bullae and H&E slides for punctured lung tissue (top ×100, bottom ×400). (b) IHC staining of 9 markers in pathological diagnosis (vimentin, SMA, desmin, PR, HMB45: ×200, D2-40: ×400, ER: ×400, CK: ×100, and Melan-A: ×100). (c) Sanger sequencing for mutation detection around the TSC gene mutation region.

**Table 1:** A summary of the 7 cases of male pulmonary lymphangioleiomyomatosis.

Author	Age	Immunohistochemistry	TSC
Wakida K	17	SMA (+), D2-40 (+)	Yes
Kim NR	47	SMA (+), vimentin (+), desmin (+), HMB-45 (+), PR (+), ER (−), pancytokeratin (−), epithelial membrane antigen (−)	Yes
Schiavina M	37	HMB-45 (+), ER (+), PR (+)	No
Kang HW	22	HMB-45 (+), ER (+), PR (+)	Not detected
Kabi A	18	Not detected	Yes
Yamanaka S	34	SMA (+), HMB45 (+), ER (+), PGR (+)	Yes
Wang Chunyan	76	Desmin (+), CD34 (+), D2-40 (+), SMA (+), PR (+), HMB-45 (−), Melan-A (−), ER (−)	Not detected

## Data Availability

The data generated during the present study are available from the corresponding author on reasonable request.
